# The Applicability of Provocative Functional Tests in the Diagnosis of Rotator Cuff Muscle Injuries of the Best University Athletes

**DOI:** 10.1155/2022/7728277

**Published:** 2022-10-13

**Authors:** Darijan Ujsasi, Karmela Filipović, Jelena Zvekić-Svorcan, Marko Nemet, Aleksandar Đuričin, Radojka Jokšić-Mazinjanin, Slobodan Pavlović, Saša Jovanović, Boris Popović, Valdemar Štajer, Danilo Radanović, Dragan Marinković, Milan Cvetković

**Affiliations:** ^1^Faculty of Sport and Physical Education, University of Novi Sad, 21102 Novi Sad, Serbia; ^2^Specialist Ordination for Physical Medicine and Rehabilitation ArtFizio, 21000 Novi Sad, Serbia; ^3^Faculty of Medicine, University of Novi Sad, 21102 Novi Sad, Serbia; ^4^Special Hospital for Rheumatic Diseases, 21000 Novi Sad, Serbia; ^5^Institute for Emergency Medicine, 21000 Novi Sad, Serbia; ^6^Faculty of Pedagogy in Uzice, University of Kragujevac, 31000 Uzice, Serbia; ^7^Faculty of Physical Education and Sport, University of Banja Luka, 78000 Banja Luka, Bosnia and Herzegovina

## Abstract

Rotator cuff disease, external and internal impingement syndromes, low shoulder stability, various types of trauma, and overuse injuries are all related to sports activities. In order to check symptoms in patients with disability and shoulder pain, clinicians use different methods and diagnostic imaging assessment. The research is aimed at evaluating whether there is a difference between provocation function tests (PFT) and ultrasonographic (US) testing of muscles within the rotator cuff in elite collegiate athletes. Patients (*n* = 184) were recruited from university team sports selections and tested with a standardized US examination of the shoulder and five PFTs (Speed's test, Neer's test, Hawkins test, lift-off test, Yergason's test). Based on the VAS pain assessment scale, 60 subjects had some pain, which was taken for further processing in the work (124 subjects did not have the presence of pain and were excluded from further processing). The US examination was conducted using Voluson 730 apparatus, by a linear probe, with the frequency in the range of 6-12 MHz. The chi-square test showed significant differences between PFT and the occurrence of shoulder muscle tendinitis for the following variables: Speed's test and subscapularis tendinitis (*p* = 0.02) and Speed's test and infraspinatus tendinitis (*p* = 0.01); Neer test and biceps brachii caput longum tendinitis (*p* = 0.01), Neer test and supraspinatus tendinitis (*p* = 0.02) and Neer test and infraspinatus tendinitis (*p* = 0.01); lift-off test and subscapularis tendinitis (*p* = 0.05); and Yergason's test and biceps brachii caput longum tendinitis (*p* = 0.03) and Yergason's test and subscapitis tendinitis (*p* = 0.01). The greatest effect of differences was observed in Neer's test and biceps brachii caput longum tendinitis (*φ* = 0.60), while the other effects can be described as medium and small in most cases. It can be concluded that functional tests are good predictors of soft tissue changes in the muscles of the rotator cuff of the shoulder. Further monitoring and analysis are needed on a larger number of athletes.

## 1. Introduction

Rotator cuff disease is usually associated with different traumatic and mechanical causes, as well as vascular and degenerative problems. Most rotator cuff injuries are a result of the rotator cuff tendon degeneration, and this is considered to be a primary cause. However, some disorders such as smoking, steroid use, diabetes, renal disorder, and collagen-vascular disease weaken the tendon and could contribute to rotator cuff pathology. Likewise, external and internal impingement syndromes, low shoulder stability, different types of trauma, and overuse injuries are all related to athletic, sport, or occupational activity. It is one of the most common defects that can be seen in 30% of asymptomatic persons aged 60 years and over [1] and 65% of asymptomatic persons aged 70 years and over [2].

Today, athletes undertake training and participate in competition systems as the earlier generations of athletes did. Sports that require more arm strength, especially where throwing and hitting are important in the game (e.g., volleyball and handball), may cause shoulder pain more often and can lead to the occurrence of various pathological changes [3]. Some other cause, such as degenerative joint disease, glenohumeral instability, calcific tendinitis, cervical radiculitis, isolated acromioclavicular osteoarthritis, adhesive capsulitis, and nerve compression could have similar symptoms as subacromial impingement syndrome [4]. Injuries can be symptomatic but also asymptomatic and can be undetected in examination [5]. The joint surfaces and ligaments provide static joint stability, while dynamic stability is maintained by muscles and tendons [6], and such a great number of involved shoulder joints and their static and dynamic stability in the shoulder region require a complex examination. Furthermore, shoulder impingement syndrome is also found in the literature as rotator cuff disease or tendinopathy [7, 8].

In order to check the symptoms in patients with shoulder disability and pain, we may use various methods, and diagnostic imaging assessment is important when diagnosing soft tissue disorder management. Often, tests and protocols that are described in literature have not enough information to support their use, and a practicing clinician finds it difficult to recognize what procedure is especially useful.

A wide variety of modalities have been used to assess the rotator cuff, one of them being ultrasound assessment (US), computed tomography (CT), magnetic resonance imaging (MRI), and arthrography [9]. The advantages and utility of US are low-cost real-time imaging, nonappearance of radiation, and the dynamic examination possibility that is especially significant in the shoulder evaluation [10]. In the last decades, with various technical improvements that permit good resolution and higher Doppler signal power, US signal processing technique has become an important screening tool in the musculoskeletal structure examination. Also, this method could detect inflammation, injury, and hyperemia [11]. Moreover, clinicians repose trust in imaging data obtained from ultrasound and MRI in order to diagnose and detect rotator cuff disorders [12].

Previous research has documented over twenty-five special tests for the rotator cuff examination and several physical examination maneuvers that could isolate specific pathology of the shoulder, with widely ranging specific sensitivity [13, 14]. For several years, great effort has been devoted to sensitivity and specificity of functional prescanning test that are used in clinical practice in order to diagnose rotator cuff tears and impingement syndrome [2, 10, 12, 15–20]. Provocative functional tests frequently used in physical examinations and clinical evaluation (Speed's test, Neer's test, Hawkins test) are also available to coaches and physiotherapists at the sports field courts. Sometimes, it is not possible to make a difference between a full-thickness tear and a partial tear or tendinopathy using PFTs. Positive results of the functional tests (Neer's test, Hawkins test) can be confirmed by more detailed examinations, primarily MR and MRI in a significant correlation [21]. The two abovementioned tests have shown a significant similarity to ultrasound examinations in the diagnostic of BB tendinitis [22], while the sensitivity of the tests was absent in the diagnostic of changes in other articular cartilage and the tendon in the shoulder joint.

The validity of Yergason's test, Speed's test, and the bicipital groove point tenderness when determining biceps tendon disorder has been examined before [20]. MRI or surgical findings were used as the gold standard; however, no specific combination of tests has been reported to give a reliable positive predictive value. Moreover, to the author's best knowledge, very few publications that discuss the issue of correlation between provocation tests and US can be found available in literature. Hence, the objective of this study was to assess correlation between PFTs and US testing of the rotator cuff muscles in top-level university athletes.

## 2. Materials and Methods

### 2.1. Sample Description

A total of 184 male athletes from the University of Novi Sad, Serbia, have voluntarily participated in this study. Out of a total of 184 surveyed respondents, using the VAS pain assessment scale, 60 respondents had some pain, which were taken for further processing in the work, while 124 subjects did not have the presence of pain and were excluded from further processing.

They were also involved in different top-level university sports such as soccer, volleyball, handball, kick-boxing, dancing, and fitness, and all of them have practiced a minimum once a day, four times a week. The study was conducted according to the criteria outlined by the Declaration of Helsinki, by the ethical permission and approval from the university's Institutional Review Board (235/2-013).

### 2.2. Sample of Measuring Instruments/Variables

All the participants in the study came to a special hospital for rheumatic diseases in Novi Sad, Serbia. The US examination was conducted using Voluson 730 apparatus, by a linear probe, with the frequency in the range of 6-12 MHz. US has shown to be accurate as a diagnostic triage tool used to diagnose rotator cuff tears and soft tissue disorders [23]. The study compared the US and the MRI and found that they achieve accuracies similar in both sensitivity and specificity [23]. Ultrasound allows us to register pathological conditions of the rotator cuff not only in the painful shoulder conditions but also in asymptomatic cases. Ultrasound is particularly effective in assessing the dynamic stabilizers of the rotator cuff [24]. It is widely available, cost-effective, noninvasive, and well-tolerated [8]. The tests were used to assess long head of the biceps brachii muscle (m BB), the supraspinatus muscle (m SSP), the infraspinatus muscle (m ISP), the subscapularia muscle (m. SSB), and the teres minor muscle (m. TSM). The same doctor examined all the subjects' dominant arm, and the duration of the examination was about 20 minutes. For the purpose of processing, the results from US examination were divided into four criteria similar to the ones in Alan's [24] study:

- There are no signs of disease
- Initial signs of tendinitis
- Clear signs of tendinitis
- Clear signs of tendinitis with calcification

### 2.3. Description of the Procedure

In the case of functional provocation tests, the results are presented in the form of a dichotomous qualitative variable with two possible answers:

- Absence of pain
- Presence of pain

Before the examination, every subject's shoulder was tested using PFTs [25]:

Speed's test: to perform Speed's test, the examiner starts with the patient's arm in shoulder flexion, continues with external rotation, which is followed by full elbow extension, and finally, forearm supination; the examiner applies resistance by performing a downward movement. The test will come positive if the patient feels pain in the bicipital tendon or bicipital groove [26]

Neer's test: this test demonstrates pain during passive abduction of the arm while the scapula is stabilized. The examiner positions the arm in the scapular plane and internally rotates the arm. The test was initially described in 1977 and did not describe a painful arc. However, a painful arc that occurs in abduction is often connected with the eponym. As an addition to this maneuver, the examiner administers an injection of local anesthetic into the subacromial space and reduces the pain, which represents Neer's test. The test is positive in case a significant reduction or abolition of pain is detected [27]

Hawkins test: this test was first described in 1980, and again, it is a passive test. The examiner positions the patient's arm at 90° in the scapular plane, then bends the elbow to 90°, and passively internally rotates the arm. Pain created by this maneuver is a clear indication that the test is positive [27]

Lift-off test: the test starts with the patient lifting the dorsum of the hand to the position of the mid-lumbar spine. After that, the patient tries to lift the dorsum of the hand off of the back. The patient should be able to maximally internally rotate the shoulder, but that is not always doable due to shoulder pain or tightening of the posterior shoulder capsule. The test will come positive if the patient cannot lift the hand away from the back, or if they lift the hand by extending the shoulder or elbow. A rupture or neurological involvement can result in the absolute loss of strength, while pain inhibition or actual weakness can lead to diminished strength

Yergason's test: the patient can be in a seated or standing position, the humerus should be in a neutral position, and the elbow should be at the position of 90 degrees flexion. The patient is instructed to externally rotate and supinate their arm while the therapist manually applies resistance. Yergason's test is positive if pain is experienced in the bicipital groove during the test

### 2.4. Data Analysis

Determining the differences between the PFT and the level of tendinitis in subjects with pain (*n* = 60), which were obtained using the VAS pain scale, the parametric statistical method chi-square test was used with a level of statistical significance of *p* ≤ 0.05. In order to determine the size of the effects of the differences, the Phi indicator of the size of the effects (*φ*) was used. The classification of effects was determined according to [27]: 0.10-0.30 small effect, from 0.30 to 0.50 medium effect, and >0.50 large effect.

## 3. Results

The total sample of participants and their descriptive parameters is shown in Table 1. All the respondents are high university level athletes; all of them are in the training process and have over 9 years of experience in a specific team sport.

Table 2 shows the results of the chi-square test, which tested the significance of the differences in the distribution of the results of subjects of different groups, with the absence and presence of pain during the PFT, on certain items related to the occurrence of tendinitis of the shoulder rotator cuff muscles. The obtained results show that there is a statistically significant difference in the following variables:

1. Speed's test and tendinitis subscapularis (*p* = 0.02) and Speed's test and tendinitis infraspinatus (*p* =0.01)
2. Neer's test and biceps brachii caput longum tendinitis (*p* = 0.01), Neer's test and tendinitis supraspinatus (*p* = 0.02), and Neer's test and tendinitis infraspinatus (*p* = 0.01)
3. Lift-off test and tendinitis subscapularis (*p* = 0.05)
4. Yergason's test and biceps brachii caput longum tendinitis (*p* = 0.03) and Yergason's test and tendinitis subscapularis (*p* = 0.01)

No statistically significant differences were observed in other analyzed variables.

The greatest effect of differences is noticeable in Neer's test and biceps brachii caput longum tendinitis of *φ* = 0.60, while the other effect can be mostly described as medium and small.

Figure 1 shows the percentage representation of subjects with and without pain in Speed's functional test in the presence of subscapularis tendinitis. Significant differences between Speed's test and subscapularis tendinitis variables were observed (*p* = 0.02; *χ*^2^ = 5.88). According to Cohen [28], the medium effect of differences was observed (*φ* = 0.31). Initial signs of tendinitis were observed in 30.8% of subjects with pain and 6.4% of subjects without pain.

Figure 1 shows the frequencies of the results for subjects with and without pain in Speed's functional test in the presence of infraspinatus tendinitis. The results indicate significant differences between the variables Speed's test and infraspinatus tendinitis (*p* = 0.02; *χ*^2^ = 19.81). According to Cohen [28]. the large effect of differences was observed (*φ* = 0.58). Clear signs of tendinitis are present only in 4.3% of subjects with absence of pain, while initial signs of tendinitis are present in 53.8% of subjects with presence of pain and only 4.3% of subjects with absence of pain.

There are significant differences between the two groups of subjects with and without pain and the occurrence of biceps caput longum tendinitis (*p* = 0.01) at a value of *χ*^2^ = 21.24 (Figure 2). Clear signs of tendinitis were observed in 37.5% of subjects with pain while no clear signs were observed in the group of subjects without pain (0%). Initial signs of tendinitis were observed in 17.3% of subjects without pain. A large effect of differences was observed (*φ* = 0.60) [28].

The obtained results indicate that there are significant differences between the two groups of subjects with and without pain and the occurrence of supraspinatus tendinitis (*p* = 0.02; *χ*^2^ = 9.40) (Figure 2). Clear signs of tendinitis with calcification were observed in 1.9% of subjects without pain while they were not observed in the group with pain. Clear signs of tendinitis were observed in 25% of subjects with pain and 1.9% of subjects without pain. Initial signs of tendinitis were observed in 37.5% of subjects with pain and 23.1% of subjects without pain. The effect of differences was at medium level (*φ* = 0.60) [28].

Figure 3 shows the results for subjects with and without pain in the Neer functional test with the occurrence of infraspinatus tendinitis. The obtained results indicate the existence of a significant difference (*p* = 0.01; *χ*^2^ = 8.98). The medium effect of differences was observed [28] (*φ* =0.58). Clear signs of tendinitis were observed in 3.8% of subjects without pain, and there were no subjects with pain in this category. However, 50% of the subjects with pain had initial signs of tendinitis and only 9.6% of the subjects without pain.

The results obtained in Figure 3 show that there are significant differences (*p* = 0.05) between the two groups of subjects with and without pain in the lift-off test and the occurrence of subscapularis tendinitis at the value *χ*^2^ = 3.91. Initial signs of tendinitis were observed in 30% of subjects with pain and only 8% of subjects without pain. The correlation effect according to Cohen [28] presented and calculated using the Phi coefficient indicates a large effect (*φ* = 0.26).

The obtained results from Figure 4 show that there are significant differences between the two groups of subjects in Yergason's test with and without pain and the occurrence of biceps brachii caput longum tendinitis (*p* = 0.03, *χ*^2^ = 6.95). Initial signs of tendinitis were observed in 40% of subjects with pain and 10% of subjects without pain. Clear signs of tendinitis were observed in 10% of subjects with pain and 4% of subjects without pain. The effect of differences was at medium level (*φ* = 0.26) [28].

The obtained results from Figure 4 show that there are significant differences between the two groups of subjects in Yergason's test with and without pain and the occurrence of subscapularis tendinitis (*p* = 0.01; *χ*^2^ = 9.35). Initial signs of tendinitis were observed in 40% of subjects with pain and only 10% of subjects without pain. The correlation effect according to Cohen [28] presented and calculated using the Phi coefficient indicates a medium effect (*φ* = 0.40).

## 4. Discussion

Athletes often suffer from rotator cuff disorders, which are the cause of shoulder pain. Shoulder pain is also a common symptom in musculoskeletal clinics. There is extensive literature available [12] on special tests and other physical examination maneuvers and some of the tests described in the literature lack sufficient information to support their use. Diagnostic and evaluation procedures for detecting rotator cuff injuries and their goal to assess the extent of injuries and morphological characteristics of the same are tested daily. For this reason, the basic clinical methods and their application in everyday examinations of university-level athletes should not be neglected or denied.

The aim of the study was to evaluate the correlation between PFT and muscle testing within the US rotator cuff in elite collegiate athletes. Looking at the results, we noticed that there were significant differences between PFT and US which revealed tendinitis of the rotator cuff muscle of the dominant hand. A relationship was established between some functional tests (Speed's test, Neer's test, lift-off test, and Yergason's test) and tendinitis of the biceps brachii muscle of the long head (caput longum), tendinitis subscapularis, tendinitis infraspinatus, and tendinitis supraspinatus, as determined using US. However, it should be noted that the effects were small or medium, which could affect the final conclusions regarding the abovementioned associations between the tests and shoulder pain. Contrary to this, there is no statistically significant relationship between functional tests and the occurrence of subscapularis muscle tendinitis and infraspinatus muscle tendinitis detected by US [22].

We can say with great certainty that the mentioned provocation tests are applicable for the evaluation of pathological changes in the tendons around the long head of the biceps muscle. However, observing the pathological changes in the tetra supraspinatus, the lift-off test and the Yergason test indicated changes; so, the application of these tests is justified. This is also the case with tendinitis of the subscapularis muscle as well as the infraspinatus muscle. These facts impose an additional need to test for pathological changes using some other tests (external sign of 0-degree lag rotation, drop signal, Jobe's test (empty can test), arm drop test, abdominal pressure test, bear hug test) and diagnostic procedures [6, 17], as well as the application of magnetic resonance. Various provocative test maneuvers have been created to help identify biceps tendon lesions. The Yergason, Neer, Hawkins, and Speed tests are often used to isolate biceps tendon pathology by creating an impingement below the coracoacromial arch [29, 30].

The occurrence of tendinitis in young athletes can be explained by the excessive volume and intensity of training in younger age categories and inappropriate dosing of loads that is not in accordance with physical growth and development during long-term sports (the average number of sports participants was about 8 years), but we should not forget some changes in the soft tissues that could have occurred as a result of inadequate intake of supplements (D and K vitamins) and some hereditary or acquired diseases. These phenomena were not included during the evaluation of the external validity of the research; so, they represent a shortcoming and limitation of the research.

The advantages of using provocation tests in the diagnosis of pathological changes in the tendons of the shoulder joints are multiple. First of all, they do not require much time and practically no apparatus and, if used correctly, can be a good prescanning technique in detecting pathological changes in the rotator cuff of the shoulder. Another important advantage of provocation tests is that they can be relatively easily learned and applied in the field, outside of medical facilities. Consequently, medical professionals are not the only people who should be doing these tests, but coaches and other professional sports professionals can also use them. Although it is often enough to determine the clinical picture [16], it is necessary to be careful and to remove the suspicion of pathological changes in the shoulder joint with a more detailed medical examination. Furthermore, a physical examination protocol can be used in patients with suspected rotator cuff tears, impingement syndrome, and biceps tenosynovitis [12, 13, 16], and these are common tests and our work was to determine how much the tests helped or did not help the examiner to understand what the actual pathology of a rotator cuff injury is. The main limitation of the experiment is defining the classification of ultrasound images, reliability, and presentation of the pathology itself. Addressing this limitation, the authors suggest examining American images by a large number of professionals. Moreover, as a limitation, we must mention the strength of the correlation between the variables. Therefore, future studies should keep this in mind when designing their studies.

The results of the research indicated justified use of PFT on the muscles of the shoulder rotator cuff, especially on changes in the muscles of m. subscapularis, biceps brachii caput longum, and m. infraspinatus, because any change reduces the volume and amplitude of movement that is necessary for normal functioning. The research is even more significant since it dealt with a population of athletes, where the injuries to the muscles of this region are more pronounced than in persons who do not play sports. And any change can remove them from training and further competition, thus hampering their further careers. This study showed the presence of a set of changes that can be detected by the ultrasound and through provocative functional tests in athletes, which were more frequent in people who reported pain in the shoulder joint. Because of this, a lot of similarities can be observed with the results of other authors' research [29–32]; although, they dealt not only with athletes but also adults. The absence of any clinical sign of local pathology cannot rule out the presence of local abnormalities and constant checking of the muscles of the shoulder rotator cuff is required, since these are quite young athletes with a career ahead of them [33–35].

It should be noted that there are a lot of asymptomatic conditions in the rotator cuff muscles as well as evidence of tissue changes in people who have not even reported frequent pain [36, 37]. Our research nevertheless pointed out the importance in athletes who have reported the occurrence of pain to certain provocative functional tests, but it would be justified to conduct research on the population of people who have not reported pain in order to determine whether there might be some changes in tissues by applying ultrasound or better yet, magnetic resonance imaging. Also, in some earlier studies [38], it was pointed out that the pathology of the rotator cuff muscle was still unclear and not understood completely, and even that certain asymptomatic changes can eventually become chronic. Therefore, the thickening of the tendon, the change in the form of tendinitis, determines the duration of treatment, as well as the time of recovery that will be required for the athlete to return to training [38, 39].

Musculoskeletal shoulder adaptations can be typical for athletes; so sometimes, there are changes that are not detected by PFT but can be observed through ultrasound imaging. In our research, as well as in the research of other authors [40], such changes in tendons that have not previously been detected by PFT, namely, the thickened dominant tendon of m. subscapularis and m. biceps brachii, may also be leading risk factors for shoulder injury in athletes [29, 41, 42].

The limitation of the study is the lack of a control group of respondents, as a limited number of respondents of university age. PFTs were not compared with magnetic resonance tests, because the subjects did not feel too much pain, no connective tissue rupture was suspected nor was this expected from the aim of the study. The study was aimed at validating of the PFT in the assessment of potential shoulder rotator cuff muscle injuries. Magnetic resonance was not planned in the work methodology, because US was used as a screening method [43]. Students, if necessary, underwent MRI and were excluded from the study. It should be emphasized that US is easily available, cheaper, has no negative radiation, and is repeatable [44]. Also, the US method is used to monitor local findings, and larger partial and total ruptures can be seen; so, a differential diagnosis can be made in relation to inflammatory rheumatic diseases.

## 5. Conclusions

Certain differences in the manifestation of tendinitis were found in athlete subjects who reported pain. Based on the obtained and presented research results, it can be concluded that PFTs are good indicators of changes in soft tissues and different degrees of damage, and that they can be used as initial indicators of these conditions. Knowledge of common locations of this condition, for rotator cuff tendons, can enable focusing medical examinations and increase the sensitivity of this field of work of sports and medical workers.

## Figures and Tables

**Figure 1:** Functional Speed's test and subscapularis tendinitis and functional Speed's test and infraspinatus tendinitis.

**Figure 2:** Neer test and biceps brachii caput longum tendinitis and functional Neer test and supraspinatus tendinitis.

**Figure 3:** Functional Neer test and infraspinatus tendinitis and functional lift-off test and subscapularis tendinitis.

**Figure 4:** Functional Yergason's test and biceps brachii caput longum tendinitis and functional Yergason's test and subscapularis tendinitis.

**Table 1:** Participants' characteristics.

*n* = 60	*M* ± SD
Age (years)	22.21 ± 1.64
Height (cm)	180.84 ± 8.21
Weight (kg)	75.20 ± 9.41
Sports experience (years)	8.72 ± 3.99
Practiced a day (1-3 times per week)	1.13 ± 0.39
Practiced a week (3-6 times per week)	4.76 ± 1.40
Shoulder injuries (*n*)	48
Pain in shoulder (VAS scale) (*n*)	60
Speed's test (*n*)	14
Neer's test (*n*)	9
Hawkins test (*n*)	41
Lift-off test (*n*)	11
Yergason's test (*n*)	15

Legend: *M*: arithmetic mean; SD: standard deviation; *n*: number of cases.

**Table 2:** Results of the differences between subjects with the presence and absence of pain in PFT and the occurrence of tendinitis of the shoulder rotator cuff muscles.

	Biceps brachii caput longum tendinitis (*n* = 16)	Tendinitis subscapularis (*n* = 12)	Tendinitis supraspinatus (*n* = 31)	Tendinitis infraspinatus (*n* = 17)
Speed's test				
*χ*^2^ (df)	3.82 (2)	5.88 (1)	6.25 (3)	19.81 (2)
*p* (*φ*)	0.15 (0.25)	0.02 (0.31)	0.10 (0.32)	0.01 (0.58)
Neer's test				
*χ*^2^ (df)	21.24 (2)	1.59 (1)	9.40 (3)	8.98 (2)
*p* (*φ*)	0.01 (0.60)	0.21 (0.16)	0.02 (0.40)	0.01 (0.39)
Hawkins test				
*χ*^2^ (df)	3.43 (2)	3.02 (1)	6.42 (3)	4.91 (2)
*p* (*φ*)	0.18 (0.24)	0.08 (0.22)	0.09 (0.33)	0.09 (0.29)
Lift-off test				
*χ*^2^ (df)	5.75 (2)	3.91 (1)	1.04 (3)	2.00 (2)
*p* (*φ*)	0.06 (0.31)	0.05 (0.26)	0.79 (0.13)	0.37 (0.18)
Yergason's test				
*χ*^2^ (df)	6.95 (2)	9.35 (1)	0.93 (3)	2.69 (2)
*p* (*φ*)	0.03 (0.34)	0.01 (0.40)	0.82 (0.12)	0.26 (0.21)

Legend: *χ*2: chi-square test value; *p*: level of statistical significance chi square test; df: degrees of freedom; *φ*: Phi coefficient of effects.

## Data Availability

Data will be available from the corresponding author if required.
